# Effects of Nucleotides Supplementation of Infant Formulas on Plasma and Erythrocyte Fatty Acid Composition: A Meta-Analysis

**DOI:** 10.1371/journal.pone.0127758

**Published:** 2015-06-23

**Authors:** Lanfang Wang, Jing Liu, Huan Lv, Xingwei Zhang, Li Shen

**Affiliations:** 1 Institute of Nutrition and Healthy Food, Tongji University School of Medicine, Shanghai, China; 2 Department of Pathogen Biology, Tongji University School of Medicine, Shanghai, China; Northwestern University Feinberg School of Medicine, UNITED STATES

## Abstract

**Objective:**

Nucleotides (NTs) have been added to infant formulas for several years due to their health benefits. However, studies have reported inconsistent findings regarding the association between NTs and fatty acid (FA) composition. A meta-analysis was performed to assess the effects of NTs supplementation of infant formula on erythrocyte and plasma FA composition.

**Methods:**

Randomized controlled trials that evaluated the association between NTs supplementation and FA composition and were published before October 2014 were included. Standardized mean differences (SMDs) with 95% confidence intervals (CIs) were calculated. Heterogeneity was assessed using Q and *I* ^2^ tests.

**Results:**

Eight studies (364 infants) were included in the meta-analysis. NTs supplementation did not affect the concentrations of total saturated FAs (SMD= 0.05; 95% CI= -0.23–0.32; *P* = 0.75) or total monounsaturated FAs (SMD= -0.01; 95% CI= -0.28–0.27; *P* = 0.95) in erythrocyte membranes. Erythrocyte total n-3 (SMD= 0.15; 95% CI= -0.11–0.41; *P* = 0.27) and n-6 PUFA (SMD= -0.16; 95% CI= -0.42–0.10, *P* = 0.22) concentrations did not increase with NTs supplementation. The concentrations of erythrocyte n-3 PUFA (18:3, 20:5, 22:5, and 22:6) and n-6 PUFA (18:2, 20:3, 20:4, and 22:4) were not affected by NTs supplementation. NTs significantly increased plasma concentrations of 18:2 n-6 (SMD= 0.90; 95% CI= 0.47–1.33; *P* < 0.0001), 20:3 n-6 (SMD= 0.56; 95% CI= 0.14–0.97; *P* = 0.009), and 20:4 n-6 PUFA (SMD= 0.92; 95% CI= 0.50–1.35; *P* < 0.0001), and significantly decreased the concentration of plasma 18:3 n-3 PUFA (SMD= -0.60; 95% CI -1.12 to -0.09; *P* = 0.02). No effect was obtained on plasma 20:2 n-6 PUFA concentrations (SMD= 0.06; 95 % CI, -1.03 to -0.2; *P* = 0.93).

**Conclusions:**

Our meta-analysis revealed that NTs supplementation significantly increased plasma 18:2 n-6, 20:3 n-6, and 20:4 n-6 PUFA concentrations in infants, but did not affect erythrocyte FA composition.

## Introduction

Nucleotides (NTs), which are non-protein, nitrogenous compounds that participate in biological processes, are considered to be conditionally essential nutrients during infancy [1]. Human milk contains higher amounts of NTs compared to bovine milk; therefore, NTs have been added to bovine milk-derived infant formulas for several years [2, 3]. NTs have beneficial effects on early infant growth [4, 5], small intestinal growth and development [6–8], intestinal microflora [9], and immune function [10, 11].

It has been reported that NTs increase the levels of long-chain polyunsaturated fatty acids (LCPUFA) in infants. According to some studies, NTs supplementation in infant formulas increases LCPUFA concentrations in erythrocyte membranes and plasma phospholipids in infants [12, 13]. Total n-6 and n-3 LCPUFA concentrations are similarly increased by NTs supplementation [12, 14]. However, more recent studies have not confirmed the beneficial effects of NTs on erythrocyte fatty acid (FA) composition [15–18]. LCPUFA are important in infant growth and development, especially docosahexaenoic acid (DHA, 22:6 n-3) and arachidonic acid (ARA, 20:4 n-6) [19]. Therefore, the interaction between NTs and LCPUFA may be of importance in infant nutrition. In this study, we performed a meta-analysis to evaluate whether NTs supplementation in infant formulas affects FA composition.

## Methods

### Ethics statement

We performed a meta-analysis of published randomized controlled trials (RCTs) assessing the effects of NTs supplementation of infant formula on erythrocyte and plasma FA composition. The analyses have been approved by the Ethics Committee of Tongji University. Parents of infants enrolled in published RCT studies have provided written informed consent before any study-related procedure was performed.

### Search strategy

A systematic literature search was performed using PubMed, Web of Science, OVID-MEDLINE, Cochrane Library, China Knowledge Resource Integrated Database, and Wanfang Database to identify relevant studies published in English and Chinese through October 2014. The search terms were the following, “formula” and “nucleotides”, “ribonucleotides”, “nucleosides”, or “ribonucleosides”. The human subjects were limited to infants. A manual search of references from related articles was also performed.

### Inclusion criteria

The inclusion criteria of our meta-analysis were (1) randomized controlled trials (RCTs) assessing infant formulas with and without NTs supplementation, (2) RCTs assessing infant FA concentrations as an outcome, (3) NTs supplementation initiated within one month post-birth, and (4) FA concentrations expressed as mean ± SD (or ± SE).

### Data extraction and study quality assessment

Two investigators independently extracted data (e.g., first author’s name, year of publication, country of origin, start and duration of supplementation, and sample size) from the RCTs. Discordances were discussed and resolved. Where data were incomplete, we contacted the corresponding authors and asked for relevant information.

Study quality was assessed using the Jadad scale [20], which evaluates studies based on three aspects: method of randomization, adequacy of blinding, and completeness of follow-up. The minimum and maximum assigned scores were 1 and 5, respectively. RCTs with 1–2 and 3–5 scores were considered to be low and high quality, respectively.

### Statistical analyses

Our meta-analysis was performed using Cochrane RevMan 5.2 software (The Nordic Cochrane Centre, Copenhagen, Denmark). For each study, standardized mean differences (SMDs) with 95% confidence intervals (CIs) for continuous data were calculated. Statistical heterogeneity among studies was assessed using Q and *I* ^2^ tests; heterogeneity was considered significant at *P <* 0.10 or *I* ^2^ > 50%. A fixed-effects model was used when there was no significant heterogeneity among studies; alternatively, a random-effects model was used.

## Results

### Characteristics of studies and quality assessment

A total of 222 studies were obtained in the primary search, of which 212 studies were excluded based on the title and abstract (Fig 1). Among the remaining 10 studies, two were excluded because one study was not an RCT [21] and one study had no sufficient information [22]. A total of eight studies were included in the meta-analysis [12–18, 23]. Of these studies, six studies reported the effect of NTs on erythrocyte FA concentrations [13–18]; three studies reported the effect of NTs on plasma FA composition [12, 18, 23].

**Fig 1:** Flow chart of literature search and study selection procedure. RCT: randomized controlled trial.

The characteristics of the eight studies are shown in Table 1. In total, 364 infants were included in the meta-analysis. The initiation of NTs supplementation was within one and a half months post-birth. The studies were conducted in Spain, Sweden, Netherlands, Italy, and Australia between 1986 and 2005. Study duration ranged from 4 weeks to 7 months. Two studies reported increased contents of plasma n-6 and n-3 PUFA after NTs supplementation of infant formulas [12, 23]. One study reported favorable effects of NTs on erythrocyte phosphatidylethanolamine and phosphatidylserine levels [14], whereas five studies did not show any significant effects on erythrocyte LCPUFA concentrations [13, 15–18].

**Table 1:** Characteristics of included studies.

Author	Year	Number	Country	Infants	Initiation (post-birth)	Duration	Jadad Scale	Nucleotides (mg/L)
Gil et al.	1986	58	Spain	Term	0 day	4 weeks	1	18.97
DeLucchi et al.	1987	38	Spain	Term	0 day	30 days	2	18.97
Gil et al.	1988	38	Spain	Term	0 day	4 weeks	2	18.97
Pita et al.	1988	36	Spain	Preterm	0 day	30 days	2	21.85
Woltil et al.	1995	68	Netherlands	Low-birth-weight	11 ± 2 days	31 days	3	11.70
Axelsson et al.	1997	26	Italy	Preterm	0 day	6–7 weeks	2	37.60
Hernell et al.	2002	22	Sweden	Term	4 ± 2 weeks	5 months	3	40.00
Gibson et al.	2005	136	Australia	Term	0 day	7 months	5	33.50

The quality scores of each study are shown in Table 1. The quality scores ranged from 1 to 5. Out of the eight studies, three were of high quality (scores >2), while the remaining five studies were of low quality (scores ≤2).

### Effect of NTs on erythrocyte FA composition

Six studies including 288 infants evaluated erythrocyte FA composition. As shown in Fig 2, NTs supplementation did not affect total saturated FA (SMD = 0.05; 95% CI = -0.23–0.32; *P* = 0.75; *I* ^2^ = 0%) or total monounsaturated FA (SMD = -0.01; 95% CI = -0.28–0.27; *P* = 0.95; *I* ^2^ = 0%). The concentrations of total n-3 (SMD = 0.15; 95% CI = -0.11–0.41; *P* = 0.27; *I* ^2^ = 0%) and n-6 PUFA (SMD = -0.16; 95% CI = -0.42–0.10; *P* = 0.22; *I* ^2^ = 0%) were not affected in the NTs supplemented group.

**Fig 2:** Forest plot of nucleotides supplementation and erythrocyte fatty-acid contents. CI: confidence interval.

NTs supplementation had no effects on 18:3 n-3 PUFA (SMD = 1.06; 95% CI = -0.49–2.61; *P* = 0.18), 20:5 n-3 PUFA (SMD = -0.01; 95% CI = -0.27–0.25; *P* = 0.91), 22:5 n-3 PUFA (SMD = 0.03; 95% CI = -0.33–0.40; *P* = 0.86), or 22:6 n-3 PUFA (SMD = 0.08; 95% CI = -0.15–0.31; *P* = 0.51) concentrations (Fig 3). The results showed that the overall concentrations of erythrocyte n-6 PUFA (18:2, 20:3, 20:4, and 22:4) were not affected by NTs supplementation (Fig 4).

**Fig 3:** Forest plot of nucleotides supplementation and erythrocyte n-3 PUFA contents. CI: confidence interval.

**Fig 4:** Forest plot of nucleotides supplementation and erythrocyte n-6 PUFA contents. CI: confidence interval.

There was significant heterogeneity among the studies in erythrocyte 18:3 n-3 PUFA concentrations (*I* ^2^ = 94%; *P* < 0.00001). To explore the heterogeneity among the studies, we performed a sensitivity analysis (Fig 5). The results revealed that the study by Pita et al [13] was the key contributor to the heterogeneity observed among the studies. When this study was excluded, there was no heterogeneity (*P* = 0.83; *I* ^2^ = 0%) and the pooled SMD was -0.03 (95% CI = -0.39–0.34; *P* = 0.88).

**Fig 5:** Sensitivity analysis of studies evaluating the effects of nucleotides supplementation on erythrocyte 18:3 PUFA content. CI: confidence interval.

### Effect of NTs on plasma FA composition

Three studies reported the effects of NTs supplementation on plasma FA composition; however, the method used to assess plasma FA composition in one study [14] differed from the method used in the other two studies [12, 23]. Therefore, only two studies were included in our meta-analysis [12, 23]. The results revealed that the concentrations of plasma 18:2 n-6 PUFA (SMD = 0.90; 95% CI = 0.47–1.33; *P* < 0.0001; *I* ^*2*^ = 0%), 20:3 n-6 PUFA (SMD = 0.56; 95% CI = 0.14–0.97; *P* = 0.009; *I* ^*2*^ = 0%), and 20:4 n-6 PUFA (SMD = 0.92; 95% CI = 0.50–1.35; *P* < 0.0001; *I* ^*2*^ = 0%) were significantly higher in NTs-supplemented infants (Fig 6). On the other hand, the concentration of 18:3 n-3 PUFA (SMD = -0.60; 95% CI, -1.12 to -0.09; *P* = 0.02; *I* ^*2*^ = 33%) was significantly lower with NTs supplementation. No statistically significant differences were obtained in plasma 20:2 n-6 PUFA concentration (SMD = 0.06; 95% CI, -1.34 to -0.47; *P* = 0.93; *I* ^*2*^ = 91%) between infants fed NTs-supplemented formulas and infants fed NTs-free formulas (Fig 6).

**Fig 6:** Forest plot of nucleotides supplementation and plasma PUFA composition. CI: confidence interval.

## Discussion

Our meta-analysis showed that NTs supplementation of infant formulas did not affect total saturated FA, total monounsaturated FA, total or individual n-3 PUFA, or n-6 PUFA concentrations in erythrocyte membranes. Even though Gibson et al [17] reported that NTs supplementation did not affect erythrocyte LCPUFA concentrations in late infancy (7 months of age), the authors did not exclude the possibility that NTs may affect FA composition at an earlier age or that the effect may be transitory. Hernell and Lonnerdal [16] reported that NTs had no effects on erythrocyte LCPUFA concentrations and explained that NTs concentration was lower than that required for LCPUFA synthesis [16]. Pita et al [13] reported that the concentrations of erythrocyte n-6 PUFA (20:3, 20:4, 22:4, and 22:5) were significantly lower in infants fed control formula (i.e., not supplemented with NTs) compared to human milk-fed infants, while no significant differences were observed between the NTs-supplemented and the human milk-fed groups. Pita et al suggested that NTs supplemtation may result in a better adaptation of milk formula [13].

In contrast with the results of erythrocyte FA composition, our meta-analysis revealed that NTs supplementation significantly increased the plasma content of 18:2 n-6, 20:3 n-6 and 20:4 n-6 PUFA and significantly decreased the plasma content of 18:3 n-3 PUFA. Our results were supported by animal and epidemiological studies which have shown that NTs-supplemented diets significantly increase plasma concentrations of n-6 PUFA [12, 24–26]. LCPUFA, particularly DHA and ARA, are critical for infant health and neurodevelopment [19, 27–29]. The concentration of DHA and ARA declines rapidly after birth [30, 31] and low ARA is associated with poor clinical outcomes, such as an increased risk of late-onset sepsis [30]. Adequate ARA is necessary for optimal growth and cognition [31]. However, the infant has a limited ability to convert essential precursor FAs to DHA and ARA, due to reduced levels and activity of desaturase enzymes [32–34]. Studies indicated that dietary NTs play important roles in activating desaturase enzymes involved in the conversion of essential FAs to LCPUFA, resulting in ARA and DHA contents similar to those of breast-fed infants [14, 15, 23]. Our results suggest that NTs-supplementation has plasma LCPUFA-enhancing effects compared with unsupplemented formula, especially ARA. In our meta-analysis, only two studies were used to assess the association between NTs supplementation and plasma PUFA concentrations [12, 23]. These two studies originated from the same research department, thereby possibly introducing bias in our analysis. Any conclusion from these results has to be drawn with caution.

Certain limitations should be considered when interpreting the results of our meta-analysis. First, only studies published in English and Chinese were included in our meta-analysis. Studies published in other languages were excluded. Second, the supplemented levels of NTs in the eight studies ranged from 11.7 mg/L to 40 mg/L; this wide range may have affected the response to the intervention. However, carrying out a dose-response analysis of NTs and FA composition was not possible because of the limited number of RCTs in our meta-analysis. Third, the duration of NTs supplementation was short, i.e., from 4 weeks to 7 months. Therefore, we were unable to evaluate the effect of long-term supplementation in this analysis. Fourth, the RCTs included in the meta-analysis were mainly conducted in Europe and Australia; therefore, the extrapolation of the results to other populations should be performed with caution. Finally, methodological differences, confounding factors, and biases may have affected our results.

## Conclusion

The results of our meta-analysis showed that NTs supplementation significantly increased plasma concentrations of 18:2 n-6, 20:3 n-6, and 20:4 n-6 PUFA, but had no effects on erythrocyte FA content. RCTs with long-term NTs supplementation should be evaluated to reach definitive conclusions.
